RETRACTED

# Diagnostic Value of Serum Heparin Binding Protein, Blood Lactic Acid Combined with hs-CRP in Sepsis and Its Relationship with Prognosis

**DOI:** 10.1155/2021/5023733

**Published:** 2021-11-09

**Authors:** Hongsong Ma, Huasheng Liu, Changyu Wu, Lieping Huang

**Affiliations:** ^1^Department of Clinical Laboratory, Zhoushan Women and Children Hospital, Zhoushan, Zhejiang 316000, China; ^2^Department of Infectious Disease, Zhoushan Women and Children Hospital, Zhoushan, Zhejiang 316000, China; ^3^Department of Internal Medicine, Zhoushan Women and Children Hospital, Zhoushan, Zhejiang 316000, China; ^4^Department of Pediatrics, Zhoushan Women and Children Hospital, Zhoushan, Zhejiang 316000, China

## Abstract

**Objective:**

To explore the diagnostic value of serum heparin binding protein (HBP), blood lactic acid (Lac) combined with high-sensitivity C- reactive protein (hs-CRP) in sepsis and its relationship with prognosis.

**Methods:**

The clinical data of 127 patients with sepsis from March 2019 to March 2021 in our hospital were retrospectively analyzed. 120 outpatients undergoing physical examination in the same period in our hospital were selected as the control group. According to the severity of the disease, 127 sepsis patients were divided into the mild sepsis group (*n* = 45), severe sepsis group (*n* = 53), and septic shock group (*n* = 29). According to the clinical prognosis, the patients were divided into the survival group (*n* = 96) and death group (*n* = 31). Serum HBP, Lac, and hs-CRP levels were measured in all subjects. The ROC curves of the subjects were drawn to analyze the predictive value of serum HBP, Lac, and hs-CRP for the prognosis of sepsis patients.

**Results:**

The levels of serum HBP, Lac, and hs-CRP in the sepsis group were higher than those in the control group (*P* < 0.05). With the increase of the severity of sepsis, serum HBP, Lac, and hs-CRP levels of patients gradually increased (*P* < 0.05). The levels of serum HBP, Lac, and hs-CRP in the death group were higher than those in the survival group (*P* < 0.05). The AUC of serum HBP, Lac, and hs-CRP for predicting the prognosis of sepsis patients was 0.858 (95% CI: 0.763–0.953), 0.694 (95% CI: 0.589–0.799), and 0.843 (95% CI: 0.759–0.927). The AUC of serum HBP, Lac combined with hs-CRP for predicting the prognosis of sepsis patients was 0.961 (95% CI: 0.000–1.000).

**Conclusion:**

The levels of serum HBP, Lac, and hs-CRP in patients with sepsis were significantly increased and increased with the severity of sepsis. Serum HBP, Lac, and hs-CRP have a good value in predicting the prognosis of patients with sepsis and worthy of clinical application.

## 1. Introduction

Sepsis is a systemic inflammatory response syndrome that causes pathophysiological changes of the immune system due to pathogen infection and has become a common critical illness in the clinic [1]. The condition of sepsis is dangerous and progresses rapidly. If it is not treated with timely and appropriate intervention, the condition will further deteriorate, and even there will be a life-threatening multiorgan dysfunction syndrome, which has posed a serious threat to the life safety of patients [2]. Although significant advances have been made in medical technology in recent years and technologies such as antimicrobial therapy, antiinfection treatment, ventilator support, and blood purification have been widely used in clinical practice, the mortality rate of sepsis patients is still high, which can be as high as 30–50% [3]. Studies have shown that sepsis is still the main factor for the death of noncardiac patients in intensive care units [4]. Early detection of sepsis and timely and effective intervention have a positive effect on the remission and prognosis improvement of sepsis patients, which are the keys to reduce the mortality of sepsis. Bacteriology is an important reference for the diagnosis of sepsis, and the most common pathogenic factors are Gram-positive and Gram-negative bacteria. However, the success rate of blood bacterial culture is affected by many factors, and the time-consuming bacteriological examination is long, which is easy to delay the condition and increase the risk of death of patients. Therefore, it is very important to use rapid laboratory indicators to assist in the diagnosis of sepsis.

RETRACTED

Heparin binding protein (HBP), a multifunctional protein, has bactericidal and chemotactic properties, which can chemotactic and activate mononuclear/macrophage cells in the body, enhance inflammatory response, strengthen tissue damage, and microcirculation disorder. These characteristics are related to the strong positive charge of HBP itself [5]. HBP can activate endothelial cells, induce vascular leakage and tissue edema, and participate in the regulation of apoptosis. High level of HBP may lead to severe vascular leakage and inflammatory cell chemotaxis [6]. At present, studies have shown that HBP plays a role in the early diagnosis of infectious diseases such as urinary tract infection and local skin infection [7]. Blood lactic acid (Lac) is an intermediate product of the glucose metabolism produced by brain tissue, striated muscle, and red blood cells, and its level is closely related to the tissue perfusion of the body and the state of cellular hypoxia [8]. When the cells in the body lack oxygen or need a large amount of energy supply for a short time, the cells will increase the anaerobic metabolism to quickly provide an energy source. Red blood cells can only undergo anaerobic glycolysis, and almost all tissues can produce Lac. After Lac production, it is mainly metabolized by the liver and kidney. If the production rate of Lac exceeds the removal rate, it will cause the accumulation of Lac and lead to the occurrence of hyperlactatemia [9]. C-reactive protein (CRP), a marker of inflammatory response, is currently a commonly used diagnostic indicator of sepsis, with high sensitivity but lack of specificity. High-sensitivity CRP (hs-CRP) is an ultrasensitive detection technology used in clinical laboratories for accurately detecting low concentrations of CRP. hs-CRP is an acute phase inflammatory response protein secreted by liver cells under the action of interleukin-6, and its level in the serum is increased under stress conditions, thus accurately reflecting the inflammatory response state of the body [10].

RETRACTED

At present, clinical studies on the diagnostic value and prognostic value of serum HBP, Lac, hs-CRP, and the combination of the three in sepsis are relatively rare. On account of this, we explored the value of serum HBP, Lac, and hs-CRP in the diagnosis of sepsis and the evaluation of prognosis in patients, in order to provide reference for clinical diagnosis and treatment.

## 2. Methods

### 2.1. General Information

The clinical data of 127 patients with sepsis from March 2019 to March 2021 in our hospital were retrospectively analyzed. Among them, 59 cases were pulmonary infection, 24 cases were abdominal infection, 20 cases were urinary system infection, 13 cases were bloodstream infection, and 11 cases were other infections. Inclusion criteria: sepsis was diagnosed clinically; all sepsis patients were treated systematically according to the guidelines [11]; age 25–71 years old; no antibiotic treatment before admission; clinical data were completed. Exclusion criteria: severe liver diseases such as liver cancer and liver cirrhosis; leukemia, aplastic anemia; advanced malignant neoplastic disease; diseases of the blood system; women who are pregnant or breastfeeding; dropout from the study; incomplete clinical data. In addition, 120 outpatients undergoing physical examination in the same period in our hospital were selected as the control group.

According to the severity of the disease, 127 sepsis patients were divided into the mild sepsis group (*n* = 45), severe sepsis group (*n* = 53), and septic shock group (*n* = 29). Grouping criteria: (1) mild sepsis group: suspected or definite infection, with the following manifestations: systemic manifestations including hypothermia, fever, accelerated breathing, increased heart rate, change of consciousness, hyperglycemia, and obvious edema; abnormal inflammatory response indexes such as procalcitonin, hs-CRP, and white blood cell count; heart index >3.5 min/m^2^, mixed venous oxygen saturation >0.7, hypotension; abnormal tissue perfusion parameters; organ dysfunction. (2) Severe sepsis group: patients who met the diagnostic criteria of sepsis and complicated with organ dysfunction manifestations. (3) Sepsis shock group: urine volume was relatively small; hyperlactatemia; skin speckles or cold limbs; capillary refill time >2 s; hypotension.

RETRACTED

According to the clinical prognosis, the patients were divided into the survival group (*n* = 96) and death group (*n* = 31). Survival group: the patients who had reached the diagnostic criteria for sepsis in the past. After treatment in ICU, the patient's condition eased, and they were transferred to other departments for further treatment or discharged from hospital. Death group: patients who met the diagnostic criteria for sepsis in the past and died from sepsis in the hospital.

There were no significant differences in gender and age among different groups (*P* > 0.05), indicating that they were balanced and comparable, as given in Table 1.

### 2.2. Research Methods

2 mL of peripheral venous blood of patients in the control group and sepsis group was collected, centrifuged for 20 min, and the serum was stored in a −80 C refrigerator. Serum HBP, Lac, and hs-CRP levels were measured in all subjects after passing the indoor quality control. The HBP level was determined with the enzyme-linked immunosorbent assay (ELISA), Lac level was determined with the enzyme electrode method, and hs-CRP level was determined with immunoturbidimetry.

### 2.3. Statistical Methods

SPSS 22.0 statistical software was used for data processing. The measurement data of normal distribution were expressed as ($\bar{x}$ ± *s*), and comparison was performed using the *t*-test or variance test, and the enumeration data were expressed as rate (%). The *χ*^2^ test was used for comparison. For comparison between the two groups, if the distribution was normal and the variance was uniform, the *t*-test of two independent samples was adopted. For comparison among the three groups, if the distribution was normal and the variance was uniform, a one-way analysis of variance was used, and the LSD-t test was used for pairwise comparison. The working characteristics (ROC) curves of the subjects were drawn to analyze the predictive value of serum HBP, Lac, and hs-CRP for the prognosis of sepsis patients. *P* < 0.05 indicated that the difference was statistically significant. The optimal cutoff value of ROC was calculated by Youden index (Youden index = sensitivity + specificity − 1).

RETRACTED

## 3. Results

### 3.1. Comparison of Serum HBP, Lac, and hs-CRP in the Control Group and the Sepsis Group

The levels of serum HBP, Lac, and hs-CRP in the sepsis group were higher than those in the control group (*P* < 0.05), as given in Table 2.

### 3.2. Comparison of Serum HBP, Lac, and hs-CRP in Sepsis Patients with Different Conditions

With the increase of the severity of sepsis, serum HBP, Lac, and hs-CRP levels of patients gradually increased (*P* < 0.05), as given in Table 3.

### 3.3. Comparison of Serum HBP, Lac, and hs-CRP in the Survival Group and the Death Group

The levels of serum HBP, Lac, and hs-CRP in the death group were higher than those in the survival group (*P* < 0.05), as given in Table 4.

### 3.4. The Predictive Value of Serum HBP, Lac, and hs-CRP on the Prognosis of Patients with Sepsis

The AUC of serum HBP, Lac, and hs-CRP for predicting the prognosis of sepsis patients were 0.858 (95% CI: 0.763–0.953), 0.694 (95% CI: 0.589–0.799), and 0.843 (95% CI: 0.759–0.927). The AUC of serum HBP, Lac combined with hs-CRP for predicting the prognosis of sepsis patients was 0.961 (95% CI: 0.000–1.000), as given in Table 5 and Figure 1.

## 4. Discussion

Sepsis is an uncontrolled inflammatory reaction of the immune system against infection and injury, with a high risk of death, aggravating the economic burden of patients and families and seriously affecting the quality of life of patients. The clinical manifestations and progression of sepsis are not only affected by the pathogenic bacteria but also closely related to patients' age, genetic factors, environmental factors, and other factors [12]. At present, the white blood cell count is the most commonly used indicator to determine the presence or absence of infection, but it is greatly affected by individual differences and is easily affected by other factors, such as acute bleeding and myocardial infarction, and can only be used as a reference indicator. In addition, traditional indicators such as the percentage of neutrophils lack specificity and cannot accurately diagnose and evaluate the prognosis of patients with sepsis. Therefore, finding effective biological indicators for diagnosis and prognosis evaluation has become a hot topic and difficult problem in critical illness medical research.

HBP is a secretory protein released after neutrophil activation, which can participate in a variety of physiological reactions in the body. HBP concentration in healthy people is relatively low. Once the body is infected, it can activate a large number of white cells, stimulate the production of HBP, and significantly increase the concentration of HBP in blood [13]. HBP has antibacterial and chemotactic properties, and it can chemotactic monocytes, neutrophils, and T lymphocytes, increase vascular permeability, induce blood leakage to the tissue space, and intensify the inflammatory response of the body. It plays an important role in the occurrence and development of sepsis. At the same time, HBP is one of the most important upstream signals acting on endothelial cells, which is easy to contact with vascular endothelial cells, quickly activates intracellular Ca^2+^, and produces actin tension fibers, causing leakage of the paracellular pathway, thus leading to endothelial cell dysfunction and capillary leakage and other reactions, causing coagulation dysfunction and imbalance of systemic inflammatory response, further aggravating the deterioration of sepsis. In our study, we found a significant increase in HBP levels in the sepsis group compared with the control group, and HBP concentrations gradually increased as sepsis progressed. The more severe the sepsis is, the higher the serum HBP level will be, resulting in vascular leakage and aggravation of inflammatory cell chemotaxis, further aggravating the tissue damage and microcirculation disorder of the body, and thus forming a vicious circle. In addition, the results of this study showed that the serum HBP concentration in the death group was significantly higher than that in the survival group. The results suggested that serum HBP levels could be used to evaluate the outcome of sepsis patients. The ROC curve showed that the AUC of serum HBP for predicting the prognosis of sepsis patients was 0.858, which also indicated that HBP had a high predictive value for the prognosis of sepsis patients. Linder's team [14] also confirmed this conclusion. They observed patients with severe sepsis and septic shock in intensive care unit and found that sepsis patients had high HBP level in a positive correlation with the severity of the disease. HBP has a positive role in the judgment and prognosis evaluation of sepsis. HBP has the advantages of simple detection, low cost, small trauma, and can make up for the deficiencies of the scoring system. It has good clinical operability and feasibility and can be widely carried out in primary hospitals. The sepsis management can be timely carried out by detecting the level of serum HBP to reduce mortality.

RETRACTED

Serum Lac level can reflect the oxygen supply and consumption levels of tissues as well as the metabolic state of the body. In the occurrence and development of sepsis, a large number of pathogenic bacteria consume oxygen in the body and the oxygen content in blood is reduced. In addition, the effective circulating blood volume of patients with sepsis is significantly reduced, which often leads to tissue hypoxia, so the serum Lac level is significantly increased. Especially in the patients with severe sepsis and septic shock, they are usually accompanied by clinical syndromes such as circulatory dysfunction, organ dysfunction, or failure, and thus, they have a higher Lac level [15]. The results of this study have shown that serum Lac levels are closely related to the occurrence and development of sepsis, and Lac can predict the prognosis of patients. In sepsis treatment guidelines [16], it can be learned that Lac has a good early warning effect on tissue hypoxia and hypoperfusion. Patients with sepsis often have hemodynamic disorders, which lead to a significant increase of Lac. When the level of Lac is abnormal, clinicians should start fluid resuscitation as early as possible to reduce the level of Lac. Khosravani's team [17] tested the Lac level of the patients at the time of admission and found that the prognosis of critical patients with hyperlactatemia is poor. When the Lac level of the patients is greater than 2 mmol/L, the mortality rate of the patients increases 1.94–10.89 times than that of the patients with less than 2 mmol/L. The dynamic changes of Lac can indicate the improvement and deterioration of the condition. However, hyperlacticaemia can be caused by many reasons such as drug use, abnormal oxygen metabolism, and genetic diseases. Therefore, in the process of clinical monitoring of Lac levels, physicians should pay attention to distinguish other types of disease.

CRP, a protein synthesized by the liver, has levels that indicate inflammation and tissue damage in the body. CRP is the main marker of inflammatory response, which can bind to microbial polysaccharides, and activate the complement system, induce the phagocytosis of phagocytes, and remove substances that stimulate the body. CRP levels in blood of healthy people are low, while CRP levels can rise rapidly when the body is in the acute phase of infection, such as bacteria, viruses, and other infections. At the same time, some noninfectious factors, such as myocardial infarction, tumor, surgery, and trauma, can also cause the increase of the CRP value. Studies have shown that during the acute phase reaction, the liver synthesis rate of CRP dramatically increases within a few hours, reaching 1,000 times the level [18]. The sensitivity of the conventional CRP detection method is relatively low, and the relatively low level of CRP cannot be detected clinically. Therefore, the use of a more sensitive hs-CRP is conducive to improving the sensitivity and accuracy of the test. hs-CRP is an acute phase protein synthesized by invasion or other inflammatory stimulation of the body, and it has been confirmed that the concentration of hs-CRP plays an important role in the diagnosis and prognosis of cardiovascular diseases [19]. The results of this study could reveal that the serum hs-CRP levels in the sepsis group were higher than those in healthy people. hs-CRP concentrations increased with the increasing severity of sepsis in patients. Serum hs-CRP levels in the death group were higher than those in the survival group. ROC analysis results showed that the AUC of serum hs-CRP for predicting the prognosis of sepsis patients was 0.843. We believe that serum hs-CRP can not only assist in the early diagnosis of sepsis but also can reflect the degree of disease progression and has a certain effect in judging the prognosis of patients with sepsis.

RETRACTED

In addition, the results of the ROC curve showed that the AUC of serum HBP, Lac, and hs-CRP combined to predict the prognosis of sepsis patients was 0.961, indicating that the combined value of the three factors to predict the prognosis of sepsis patients was more valuable. It can make up for the deficiency of single index and avoid misdiagnosis and missed diagnosis, thus improving the sensitivity and specificity of diagnosis. The combined detection of the three markers in the clinic is more conducive for clinicians to evaluate the prognosis of sepsis patients, thereby improving the accuracy of death prediction and improving the prognosis of patients.

## 5. Conclusion

The levels of serum HBP, Lac, and hs-CRP in patients with sepsis were significantly increased and increased with the severity of sepsis. Serum HBP, Lac, and hs-CRP have a good value in predicting the prognosis of patients with sepsis and worthy of clinical application. The sample size included in this study is relatively small, the results are not widely representative, and the results are interfered by therapeutic factors to a certain extent. In the future, it is necessary to increase the sample size, shift from a single-center study to a multicenter study, to reduce the bias of treatment, and further confirm the accuracy of the conclusions.

## Figures and Tables

**Figure 1:** The predictive value of serum HBP, Lac, and hs-CRP on the prognosis of patients with sepsis.

**Table 1:** Comparison of clinical data among different groups (*n*, %, $\bar{x}$ ± *s*).

Group	Number of cases	Gender		Age (years)
		Male	Female	
Control group	120	63	57	49.77 ± 9.34
Sepsis group	127	69	58	51.92 ± 8.36
*t*/*χ*^2^ value		0.083		1.908
*P* value		0.773		0.057

Mild sepsis group	45	25	20	51.57 ± 9.02
Severe sepsis group	53	27	26	51.63 ± 8.84
Sepsis shock group	29	17	12	53.02 ± 8.19
*F*/*χ*^2^ value		0.487		0.293
*P* value		0.784		0.746

Survival group	96	50	46	51.83 ± 8.71
Death group	31	19	12	52.18 ± 8.03
*t*/*χ*^2^ value		0.801		0.198
*P* value		0.371		0.843

RETRACTED

**Table 2:** Comparison of serum HBP, Lac, and hs-CRP in the control group and the sepsis group (*n*, $\bar{x}$ ± *s*).

Group	Number of cases	HBP (*μ*g/L)	Lac (mmol/L)	hs-CRP (mg/L)
Control group	120	5.06 ± 0.72	0.26 ± 0.10	1.46 ± 0.19
Sepsis group	127	77.51 ± 12.49	4.32 ± 1.58	68.29 ± 10.73
*t* value		63.436	28.092	68.21
*P* value		<0.001	<0.001	<0.001

**Table 3:** Comparison of serum HBP, Lac, and hs-CRP in sepsis patients with different conditions (*n*, $\bar{x}$ ± *s*).

Group	Number of cases	HBP (*μ*g/L)	Lac (mmol/L)	hs-CRP (mg/L)
Mild sepsis group	45	39.28 ± 5.06	2.89 ± 1.30	52.04 ± 9.62
Severe sepsis group	53	75.31 ± 8.44	4.95 ± 1.63	88.61 ± 13.38
Sepsis shock group	29	140.86 ± 21.75	5.37 ± 1.88	129.93 ± 20.62
*F* value		625.640	28.867	265.09
*P* value		<0.001	<0.001	<0.001

**Table 4:** Comparison of serum HBP, Lac, and hs-CRP in the survival group and the death group.

Group	Number of cases	HBP (*μ*g/L)	Lac (mmol/L)	hs-CRP (mg/L)
Survival group	96	63.92 ± 7.81	4.04 ± 1.58	64.31 ± 9.45
Death group	31	119.59 ± 19.03	5.16 ± 1.72	80.62 ± 12.47
*t* value		23.343	3.357	7.698
*P* value		<0.001	0.001	<0.001

**Table 5:** The predictive value of serum HBP, Lac, and hs-CRP on the prognosis of patients with sepsis.

Index	AUC	SE value	Asymptotic 95% confidence interval		Optimal cutoff value	Sensitivity (%)	Specificity (%)
			Lower limit	Upper limit			
HBP	0.858	0.048	0.763	0.953	0.565	73.6	82.9
Lac	0.694	0.054	0.589	0.799	0.439	68.8	75.1
hs-CRP	0.843	0.043	0.759	0.927	0.476	71.2	76.4
HBP + Lac + hs-CRP	0.961	0.031	0.000	1.000	0.772	85.9	91.3

## Data Availability

The data used and/or analyzed during this study are available from the corresponding author upon request.
